# Multiscale Residual Network Based on Channel Spatial Attention Mechanism for Multilabel ECG Classification

**DOI:** 10.1155/2021/6630643

**Published:** 2021-05-03

**Authors:** Shuhong Wang, Runchuan Li, Xu Wang, Shengya Shen, Bing Zhou, Zongmin Wang

**Affiliations:** ^1^School of Information Engineering, Zhengzhou University, Zhengzhou 450000, China; ^2^Cooperative Innovation Center of Internet Healthcare, Zhengzhou University, Zhengzhou 450000, China; ^3^Foreign Languages Department, Zhengzhou University of Economics and Business, Zhengzhou 450000, China

## Abstract

Automatic classification of ECG is very important for early prevention and auxiliary diagnosis of cardiovascular disease patients. In recent years, many studies based on ECG have achieved good results, most of which are based on single-label problems; one record corresponds to one label. However, in actual clinical applications, an ECG record may contain multiple diseases at the same time. Therefore, it is very important to study the multilabel ECG classification. In this paper, a multiscale residual deep neural network CSA-MResNet model based on the channel spatial attention mechanism is proposed. Firstly, the residual network is integrated into a multiscale manner to obtain the characteristics of ECG data at different scales and then increase the channel spatial attention mechanism to better focus on more important channels and more important ECG data fragments. Finally, the model is used to classify multilabel in large databases. The experimental results on the multilabel CCDD show that the CSA-MResNet model has an average F1 score of 88.2% when the multilabel classification of 9 ECGs is performed. Compared with the benchmark model, the F1 score of CSA-MResNet in the multilabel ECG classification increased by up to 1.7%. And, in the model verification on another database HF-challenge, the final average F1 score is 85.8%. Compared with the state-of-the-art methods, CSA-MResNet can help cardiologists perform early-stage rapid screening of ECG and has a certain generalization performance, providing a feasible analysis method for multilabel ECG classification.

## 1. Introduction

The mortality rate caused by cardiovascular diseases is still increasing, which has caused widespread concern in the health sector [1]. The abnormal detection of cardiovascular disease is electrocardiography (ECG), which uses electrodes placed on the skin to record the electrical activity of the heart over a period of time [2]. Abnormal ECG waveforms can reflect certain pathologies [3]. The doctor gives a clinical diagnosis result through detailed evaluation and analysis of the patient's ECG. However, the large number of ECGs collected in homes and hospitals every day may hinder doctors from reviewing the data in detail [4]. With the advent of computers and artificial intelligence technologies, more and more scholars have applied computers in the field of cardiovascular disease diagnosis, using artificial intelligence methods to predict certain diseases in order to reduce the workload of doctors.

At present, there are several categories of ECGs, such as static ECG, dynamic ECG, and ECG collected from wearable ECG equipment. Considering the monitoring time, ECG monitoring can be divided into long-term monitoring and short-term monitoring [5]. The dynamic ECG belongs to long-term monitoring, while the static ECG and the ECG obtained through the wearable ECG acquisition device are short-term monitoring. Taking into account the number of leads of the ECG, it is divided into single-lead and multilead. Most of the multileads used in hospitals are mainly 12-lead. The 12-lead ECG is more comprehensive than the 1-lead or 2-lead ECG and will cover more ECG waveform information [6]. Therefore, for some complex and changeable ECG categories, many current artificial intelligence algorithm studies have fused the signals of all 12 leads to more comprehensive ECG information, which achieves accurate automatic ECG classification.

The clinical ECG reflects the patient's heart condition over a period of time. During this period of time, there may be many different categories of abnormalities in the ECG at the same time. For example, Figure 1 shows a patient suffering from atrial premature beats (APB), premature ventricular contraction (PVC), and complete right bundle branch block (CRBBB). In the clinical diagnosis report in real life, the doctor will conduct a detailed and comprehensive review of the patient's ECG, and any abnormal waveforms and rhythms that may occur will be marked in the patient's ECG diagnosis results. This illustrates that there may be more than one heartbeat category in the patient's diagnostic results; a piece of ECG data record may correspond to multiple labels at the same time.

However, the current artificial intelligence diagnosis ECG algorithms only judge that the segment of the ECG belongs to a certain category of significant abnormality and finally ignore other general abnormal information. But this information is also a response to the patient's heart condition, and doctors can judge whether there may be other hidden heart problems based on this information. It is therefore of interest to find an efficient artificial intelligence algorithm for multilabel ECG classification. The multilabel classification is widely used in the field of target detection [7, 8] and the multilabel ECG classification is still in the early exploration stage and has not been effectively applied.

To solve the problem of multilabel ECG classification, this work presents an end-to-end deep learning model CSA-MResNet, which combines a multiscale residual network with a convolutional attention mechanism to perform nine multilabel ECG classifications on the clinical acquired China Cardiovascular Disease Database (CCDD) [9]. The main contributions of this paper are as follows: (1) A multiscale residual network CSA-MResNet model based on channel spatial attention mechanism is proposed, which classifies ECG records by extracting ECG features of different scales of convolution kernels and using the channel spatial attention mechanism to pay more attention to abnormal ECG fragments; (2) the proposed method was verified in the CCDD, and the F1 score reached 88.2%, which achieved better performance compared with benchmark methods; (3) CSA-MResNet was also tested on the HF-challenge dataset with an average *F*1 score of 85.8%, which proves that the proposed method has some generalization.

The rest of the paper is organized as follows: Section 2 briefly introduces the related works, the method is described in Section 3, Section 4 gives the experiment and results, and finally, Section 5 summarizes the full text.

## 2. Related Work

A detailed review of the patient's ECG by the clinician, mainly looking at rhythm and waveform abnormalities, requires extensive experience and medical theory, but it is time-consuming and laborious to produce a clinically experienced cardiologist. With the advent of artificial intelligence, many computer research scholars use artificial intelligence technology for abnormal judgment on ECG, which is able to greatly reduce the workload and intensity of physicians, but it is still always difficult to realize precise classification because of the diversity and individual variability of ECG data. In the past few years, research scholars have conducted many studies on ECG intelligent classification [10–12] and proposed various ECG intelligent classification methods.

In the early days when artificial intelligence was widely used in medical research, some researchers used traditional machine learning methods to classify ECG. Acharya et al. [13] first denoised the ECG signal, then extracted the nonlinear features, and finally used K-NearestNeighbor (KNN) classifier to classify normal and myocardial infarction, with an average accuracy of 98.80%. Alickovic et al. [14] used multiscale principal component analysis (MSPCA) to denoise the ECG signal and used an autoregressive (AR) model for feature extraction and examined different classifiers for comparison. The highest accuracy of the five arrhythmia categories in the MIT-BIH arrhythmia database reached 99.93%. Lin et al. [15] extracted the normalized RR interval and wavelet morphological features to classify the normal, atrial premature beats and premature ventricular contraction in the MIT-BIH arrhythmia database. Pandey et al. [16] used a set of support vector machines to classify heartbeat into four categories. Rajesh et al. [17] used intrinsic mode functions to get the final features and used the AdaBoost classifier to classify heartbeat. Although the above work achieves better results, it requires manual feature extraction, which wastes time and energy for a database with huge ECG data.

Deep learning has been widely applied to the study of ECG classification because of its characteristic ability to automatically extract data features that eliminates the steps of traditional machine learning manual extraction for automatic learning of large amounts of data. Awni et al. [4] proposed the use of an end-to-end deep neural network (DNN) to classify 12 ECG categories from single-lead electrocardiographic signals, with the mean F1 score for DNN of 0.837 exceeding the mean of 0.780 by general cardiologists. Acharya et al. [18] developed a 9-layer deep convolutional neural network that achieved F1 scores of 0.83 for the detection of five different categories of ECGs. Kamaleswaran et al. [19] identified a 13-layer convolutional neural network (CNN) model that can be used to detect four beat categories, normal sinus rhythm, AF, other abnormal rhythms, and noise on single-lead short ECG recordings, achieving an average *F*1 score of 83%. Ullah et al. [20] changed the one-dimensional time series into two-dimensional spectra by short-time Fourier transform, and the proposed deep neural network model was a two-dimensional CNN composed of four convolution layers and four pooling layers to classify eight categories of the ECG in MIT-BIH arrhythmia database with the accuracy of 99.11%. Li et al. [21] used the BiLSTM-attention model to perform five different categories of ECG classification on the MIT-BIH arrhythmia database, which effectively improved the accuracy of cardiac beat classification. Yao et al. [2] proposed attention-based time-incremental convolutional neural network (ATI-CNN) achieving 81.2% overall classification accuracy for nine ECG categories.

All of the above research has achieved high precision, but it is known from clinical experience that a single ECG recording may contain more than one disease label at the same time and that physicians give more than one diagnostic result when making an ECG diagnosis, so the above studies based on single-label ECG recording cannot meet the needs.

A subset of investigators is currently beginning to explore ECG multilabel classification. Wang et al. [22] proposed an arrhythmia detection method based on the multiresolution representation of ECG signals by taking four different deep neural networks as four channel models for ECG vector representations learning and finally performed 34 kinds of ECG classification on a multilabel HF-challenge dataset with the *F*1 score of 92.38%, all higher than the results of individual channels. Cai et al. [23] developed multi-ECGNet to identify patients with multiple cardiac diseases at the same time, with an *F*1 score of 86.3% in identifying 55 arrhythmia classifications. Sun et al. [24] proposed a novel ensemble multilabel classification model to perform 7 kinds of multilabel ECG classification on the CCDD, and the final *F*1 score was 75.2%. All of the above provided feasible analysis methods for ECG multilabel classification, but all of the above validation methods were performed on a single database, which could not reflect the generalizability of the model. Li et al. [25] proposed a model consisting of inception, GRU, and attention mechanism on a private multilabel ECG dataset for nine multilabel ECG classifications with an average *F*1 score over 88.6% and a maximum of 91.9% and also extracted the relevant category on the publicly available database PhysioNet for validation with an accuracy of 92.8% but only extracted 500 pieces of data from public databases and the results were not representative. Although the above methods accomplish multilabel ECG classification, there are still shortcomings in terms of accuracy and generalizability. Therefore, applying deep learning for multilabel ECG classification remains a challenge.

## 3. Methods

The multilabel ECG classification problem uses a deep learning model to automatically extract effective information from ECG records and predicts multiple categories for each record at the same time. In this work, the key issue is to construct an effective algorithm to classify 9 kinds of multilabel ECG signals. In response to this problem, this work proposes the CSA-MResNet architecture, which integrates the multiscale residual network and the channel spatial attention mechanism structure and can automatically extract useful information from the 12-lead ECG signal to perform multilabel ECG classification.

### 3.1. Problem Formulation

The multilabel classification task of ECG signals is to automatically classify 9 ECG categories using clinical 12-lead ECG. The proposed model requires the input of 12-lead ECG records and the output of the possible prediction labels. In the original ECG record *x*_*i*_, together with the corresponding reference label space *Y*_*i*_={*y*_1_, *y*_2_,…, *y*_*q*_},  0 ≤ *q* ≤ 8 represents a label space with *q* possible class labels, where *x*_*i*_ ∈ *ℝ*^5000×12^ is a signal with length 5000 and 12 leads. The multilabel ECG classification task is from the multilabel training set *D*={(*X*_*i*_, *Y*_*i*_)*|*1 ≤ *i* ≤ *N*} learning function *f* : *x*_*i*_⟶(*y*_1_, *y*_2_,…, *y*_*q*_), where *N* is the total number of samples, and 0 ≤ *y*_*j*_ ≤ 1,  1 ≤ *j* ≤ *q*. The output threshold is set to 0.5. If some ECG predicts that the *j*_th_ category prediction probability is greater than 0.5, then these signals are considered to belong to this *j*_th_ category, if not, otherwise. The work uses CSA-MResNet as an ECG multilabel classifier. This work uses binary cross-entropy to measure the loss between the model output and the actual sample label, as shown in

(1) $$\begin{array}{c} \mathrm{loss}\left(f\left(x_{i}\right),Y_{i}\right)=\mathrm{mean}\left(\sum_{i=1}^{q}-\omega_{i}\left(Y_{i}\times \;\log\;f\left(x_{i}\right)+{\left(1-Y\right)}_{i}\times log\left(1-f\left(x_{i}\right)\right)\right)\right), \end{array}$$

where *q* is the total number of arrhythmia categories, and 1 ≤ *i* ≤ *q*; weight *ω*_*i*_=1/log_*n*_*i*__ is the weight assigned to each category of arrhythmia; *n*_*i*_ is the number of samples of this category of arrhythmia. This allows the model to pay more attention to the categories of arrhythmias with a small number of samples, thereby reducing the impact on data imbalance to a certain extent.

### 3.2. Model Architecture

Figure 2 illustrates that the overall structure of the CSA-MResNet model is composed of a multiscale residual network and a channel spatial attention mechanism module. The network is mainly designed and constructed based on the experience of GoogleNet [26] and ResNet [27]. Both GoogleNet and ResNet are relatively mature neural networks, which can solve various image classification and target detection problems in the field of computer vision. The CSA-MResNet model contains 2 streams after the convolutional layer and the maximum pooling layer. Each stream has 32 layers of convolution and an average pooling layer, and residual connections are added on the basis of convolution to prevent the accuracy rate caused by deepening from degrading rapidly after saturation, and the channel spatial attention mechanism [28] is added before each pooling layer to obtain more important weights. The model is divided into two parts: feature fusion and multiscale feature fusion. The feature fusion includes convolution, channel spatial attention mechanism, and pooling layer. In this part, convolution is set to 15, and only the feature set of data in this scale is extracted. Then important information is filtered through the channel spatial attention mechanism, and finally the information is fused through the pooling layer. In the multiscale feature fusion part, two streams are assigned convolution kernels of different scales, which can extract convolution kernels of different scales. In each stream, a 32-layer residual network and channel spatial attention mechanism are set. Then, the features of two streams with different scales are aggregated through the pooling layer. Finally, the information on the two scales is merged and sent to the fully connected layer for 9 multilabel ECG classifications.

#### 3.2.1. Multiscale Residual Network

The multiscale residual network layer configuration is illustrated in Figure 3, where /2 means that the number of neurons passing through this layer is halved.×3,@64 represents the number of this structure multiplied by 3, and the convolution kernel number of this part is 64. (×3@64; ×4@128; ×6@256; ×3@512) is the same as the above. The main structure of this model is the residual network of two streams. The residual network is used to prevent the accuracy degradation caused by the model depth being too deep. Two streams with different scales can pay attention to the ECG features of different data segments and different leads. Finally, the features extracted from different scales of the two streams can be merged to achieve a better classification effect. One of the streams in this model is ResNet, but on the basis of its structure, the first layer of the convolutional layer and the last layer of the fully connected layer are removed, and there are 32 convolutional layers. Different convolution kernel sizes are used in the residual structure of the two streams, and the convolution kernel size of one stream is set to 3, and the convolution kernel size of the other stream is set to 7. After each convolution layer, there are a BatchNorm layer and a ReLU layer. BatchNorm [29] can speed up the convergence speed of the model, and ReLU [30] activation function can avoid gradient saturation problem.

#### 3.2.2. Channel Spatial Attention Mechanism

To better focus on abnormal ECG data, a channel spatial attention mechanism is added to the model, which can focus on channel information and spatial information at the same time, compared with the “Squeeze-and-Excitation” (SE) module that only focuses on channels [31] which has better performance. The structure is shown in Figure 4, which can combine channel information and spatial information at the same time.

The channel spatial attention mechanism includes two submodules, the channel attention mechanism (Figure 4(a)) and the spatial attention mechanism (Figure 4(b)). The channel attention mechanism obtains the channel attention map *M*_*c*_ through the selection of the channel, and in the other spatial attention mechanism to the important part of the feature of the channel, the spatial attention map *M*_*s*_ is obtained. The input feature *F* passes through these two parts to obtain the detailed feature *F*^″^. These two steps are represented by equations (2) and (3), respectively:

(2) $$\begin{array}{c} F^{\prime }=M_{c}\left(F\right)⊗F, \end{array}$$

(3) $$\begin{array}{c} F^{\prime \prime }=M_{s}\left(F^{\prime }\right)⊗F^{\prime }. \end{array}$$

Figure 4(a) shows how the channel attention mechanism works, and its ability to channel the selection of input features allows the model to focus more on channels that are useful for the task. The parameters of this module were obtained by calculating the global average pooling and the global maximum pooling information about input features, followed by merging these two parts of information, in this process both share the same fully connected network, and finally the spatial attention weights are compressed into 0-1 using the sigmoid activation function. This process can be shown as

(4) $$\begin{array}{c} M_{c}\left(F\right)=\sigma \left(MLP\left(AvgPool\right)\left(F\right)\right)+MLP\left.\left(MaxPool\left(F\right)\right)\right)\\ =\sigma \left(W_{1}\left(W_{0}\left(F_{\mathrm{avg}}^{c}\right)\right.\right)+W_{1}\left.\left(W_{0}\left(F_{\max}^{c}\right)\right)\right). \end{array}$$

Figure 4(b) shows how the spatial attention mechanism works, which can reduce the interference of other nonimportant information on the same channel to the task and improve the accuracy of the model. Features that underwent a global maximum pooling and global average pooling of features output by the channel attention mechanism were convolved, using the sigmoid activation function to compress spatial attention weights to 0-1. This process can be shown as

(5) $$\begin{array}{c} M_{s}\left(F\right)=\sigma \left(f^{1\times 7}\left(\left[\left.AvgPool\right)\left(F\right);MaxPool\left(F\right)\right]\right)\right)\\ =\sigma \left(f^{1\times 7}\left(\left[F_{\mathrm{avg}}^{s};F_{\max}^{s}\right]\right)\right). \end{array}$$

The channel attention mechanism focuses on the channels that contribute more to the ECG signal. The spatial attention mechanism assigns greater weight to more important information in different time periods of the ECG signal. The channel attention mechanism is a global application, and the spatial attention mechanism is local to the feature which plays an important role. Literature [28] shows that sequential placement has better performance than parallel placement, and the performance of channel priority is higher than spatial priority. Therefore, the attention mechanism is placed between the first convolution layer and the pooling layer and before the last pooling layer for the two streams, respectively. And the channel attention mechanism is prior to the spatial attention mechanism.

## 4. Experiments and Results

The data used in this work were obtained from a clinical 12-lead multilabel CCDD, including nine categories of ECG signals: (1) sinus arrhythmia (SA); (2) sinus bradycardia (SB); (3) T wave low and flat (TWLF); (4) sinus tachycardia (ST); (5) complete right bundle branch block (CRBBB); (6) atrial fibrillation (AF); (7) atrial premature beat (APB); (8) first-degree atrioventricular block (I-AVB); (9) premature ventricular contraction (PVC).

### 4.1. Environment

This work proposes model training and testing on XeonR Silver-4114CPU, 32 GB memory, and Geforce2080Ti graphics card. The server runs on the ubuntu 18.04 system, and the model is run on the PyTorch 1.2.0 framework.

### 4.2. Data

In this work, the CCDD multilabel dataset and HF-challenge multilabel dataset are used. In the experiment, contrasts to each indicator on different models on the CCDD are done to find the best model, followed by model generalization validation on the HF-challenge dataset. The number of ECGs used in detail is shown in Table 1.

#### 4.2.1. CCDD

The multilabel ECG samples used in this work were collected from the China Cardiovascular Disease Database [9] (CCDD). The database contains 190,000 12-lead clinical multilabel ECGs' data, the sampling rate is 500 Hz, and the data duration is 10∼20 seconds. In the CCDD, the ECG is divided into 12 primary disease types, and there are many secondary disease types. In order to make better use of the advantages of deep learning, we choose to follow the two criteria of including as many types as possible and large amounts of data. And finally this work mainly selected 9 common disease categories in the CCDD for multilabel ECG classification (when selecting data, only ECG records containing these 9 categories of labels are retained; once a label other than the above 9 types of labels appears in an ECG record, these data will be deleted). The training set and test set were divided according to the literature [32], and the validation set was randomly selected from 10% of the training set. Data processing takes 5000 points of all the ECG signals, and to ensure the quality of the signal, the first 1.25 s is discarded, and the middle 10 s data are taken. If they are less than 10 seconds, delete the data directly. The detailed data information of the final experiment can be seen in Table 1.

#### 4.2.2. HF-Challenge

The HF-challenge multilabel dataset is an ECG smart competition organized by the Tianchi platform [23]. The preliminary data contain 24106 records in the training set and 8036 in the test set A (testA), each record has 8 leads (mainly I, II and six limb lead V1∼V6), the length is 10 seconds, a total of 55 categories, the sampling rate is 500 Hz, and the unit voltage is 4.88 microvolts. This work mainly used the 9 disease categories described in Section 4.2 in the testA and expanded each piece of data to a length of 5000*∗*12 according to the official equation (6), which is Einthoven's law [33], and then multiplied by the unit voltage and converted it into real data for experiments. The ECG of cardiovascular disease may manifest in many ways. After the ECGs of different databases are marked by different doctors, the final marking description is not completely consistent due to the different degree of disease segmentation and expert marking standards, but the clinical manifestations of the disease are the same. For example, the use of flat T waves and low frequencies in the CCDD and the use of T wave changes in the HF-challenge testA are all abnormal T waveforms [34]. And the abnormal T wave is a typical manifestation of myocardial ischemia on the ECG [35]. Therefore, no distinction is made between T wave anomalies and T wave changes in this work. The distribution of the number of different categories of ECG is shown in Table 1.

(6) $$\begin{array}{c} \mathrm{III}=\mathrm{II}-\mathrm{I,}\\ \text{aVR}=-\frac{\left(I+\mathrm{II}\right)}{2},\\ \mathrm{aVL}=I-\left(\frac{\mathrm{II}}{2}\right),\\ \mathrm{aVF}=\mathrm{II}-\left(\frac{I}{2}\right). \end{array}$$

### 4.3. Training Setting

This work training uses clinical multilabel CCDD, grouping them into batches of 64 records and sending them into the model. The larger the batch, the faster the network model training, and at the same time, more memory is required. Through fine-tuning of hyperparameters, 64 were selected as the batch size. The weight initialization of the convolutional layer and the fully connected layer in CSA-MResNet uses the kaiming initializer [36] and the Adam optimizer [37] to accelerate the convergence of the network model. The default learning rate is from 0.001. In a total of 256 epochs, the learning rate is multiplied by 0.1 whenever 32, 64, and 128 epochs are encountered. The first convolution of the model is set to 15. In the two streams of the model, one of the convolution kernels is fixed at 7, and the convolution kernel size of the other stream is set differently, and the results are compared on the test set. The number of filters is performed in the order of 64, 128, 256, 512 according to different block combinations. The convolution step size of the residual connection is set to 2 to make the output size equal, and the step size of the remaining convolution and pooling is set to 1. Dropout [38] uses a ratio of 0.2 to prevent neurons from adapting to the training data. After the CSA-MResNet model is trained, the binary cross-entropy loss between the output of each batch and the actual label is calculated, and then backpropagation is performed. During the entire training period, save the model weight when the *F*1 score of the validation set is the highest.

### 4.4. Result

#### 4.4.1. Performance Metrics

This work evaluates the performance of 9 multilabel ECG classifications using the CSA-MResNet model on a large-scale test set. The work uses a multilabel classification method [39]; for the *j*_th_ class label *y*_*j*_, the four basic quantities characterizing the binary classification performance can be defined as equations (7)∼(10).

(7) $$\begin{array}{c} TP_{j}=\left|\left\{x_{i}|y_{i}\in Y_{i},y_{i}\in f\left(x_{i}\right),\;1\leq i\leq N\right\}\right|, \end{array}$$

(8) $$\begin{array}{c} FP_{j}=\left|\left\{x_{i}|y_{i}\notin Y_{i},y_{i}\in f\left(x_{i}\right),\;1\leq i\leq N\right\}\right|, \end{array}$$

(9) $$\begin{array}{c} TN_{j}=\left|\left\{x_{i}|y_{i}\notin Y_{i},y_{i}\notin f\left(x_{i}\right),\;1\leq i\leq N\right\}\right|, \end{array}$$

(10) $$\begin{array}{c} FN_{j}=\left|\left\{x_{i}|y_{i}\in Y_{i},y_{i}\notin f\left(x_{i}\right),\;1\leq i\leq N\right\}\right|, \end{array}$$

where 0 ≤ *j* ≤ 8, and *N* is the total number of samples. TP represents the number of correctly classified records of a category. FP represents the number of records that belong to other categories and are incorrectly classified into a certain category. TN represents the number of records that actually belong to other categories and are finally classified into other categories. FN refers to the number of samples belonging to a certain class that were misclassified as in other classes.

Based on the above four quantities, typical classification indicators [40–42] on each class including specificity (Spe), precision (Pre), recall (Rec), accuracy (Acc), and *F*1 score (*F*1) are derived accordingly and defined as equations (11)∼(15).

(11) $$\begin{array}{c} \mathrm{Spe}=\frac{\mathrm{TN}}{\mathrm{TN}+\mathrm{FP}}, \end{array}$$

(12) $$\begin{array}{c} \mathrm{Pre}=\frac{\mathrm{TP}}{\mathrm{TP}+\mathrm{FP}}, \end{array}$$

(13) $$\begin{array}{c} \mathrm{Rec}=\frac{\mathrm{TP}}{\mathrm{TP}+\mathrm{FN}}, \end{array}$$

(14) $$\begin{array}{c} \mathrm{Acc}=\frac{\mathrm{TP+TN}}{\mathrm{TP+TN+FP+FN}}, \end{array}$$

(15) $$\begin{array}{c} F_{1}=\frac{2\cdot \mathrm{Pre}\cdot \mathrm{Rec}}{\mathrm{Pre}+\mathrm{Rec}}. \end{array}$$

The *F*1 score is a comprehensive index with a certain degree of stability, so it is used as the final evaluation index.

#### 4.4.2. Optimal Size of Convolution Kernel

The size of the convolution kernel in deep neural networks is a key parameter that determines the performance of the model. Therefore, in this experiment, a comparison of different convolution kernel sizes is set. After the model structure is fixed, ensure that the convolution kernel size of one stream is 7, and the convolution kernel of the other stream is selected in (3, 5, 7, 9, 11), which are MResDNN-37, MResDNN-57, MResDNN-77, MResDNN-79, and MResDNN-711. For comparison to derive the most appropriate number of streams, three different convolution kernel scale sizes of MResDNN-357 were set. The above models all set the same hyperparameters such as optimizer, batch size, and learning rate. The classification results of different convolution kernel size models in the multilabel CCDD test set are shown in Table 2.

Table 2 compares the Acc, Sen, Pre, Rec, and *F*1 of different convolution kernel size models in the classification of nine multilabel ECGs. The results show that when performing multilabel abnormal ECG classification, comparing the results of MResDNN-357 with the other three models, the average *F*1 score is only 86.2%, which indicates that the classification performance of the three streams is the lowest. In the MResDNN-37, CRBBB increased by up to 3.7%, APB increased by up to 3.4%, and the final *F*1 score was also the highest among the above models, reaching 86.8%, which may be because the greater the difference in scale, the greater the degree of difference in obtaining ECG features. It can be seen from the results in the table that the final score of *F*1 of PVC and APB is lower, because the deep learning performance is greatly affected by the amount of data. PVC has fewer data pieces in the training set, and the model does not fully learn all the characteristics, while APB accounts for the largest proportion of all the data in the training set and the test set, and the data distribution affects the model performance to a certain extent. And TWFL has a low *F*1 score because of the largest proportion difference between the training set and the test set. It can better represent the more comprehensive characteristics of the ECG signal. According to the experimental results, the two convolution kernel sizes of 3 and 7 are selected as the benchmark in the two streams.

#### 4.4.3. Optimal Position of Channel Spatial Attention Mechanism

The results of Section 4.4.2 show that the best result is when the convolution kernel size of one stream is fixed to 3 and the convolution kernel size of the other stream is 7, so the channel spatial attention mechanism is embedded on this benchmark. In order to select the embedding position of the channel spatial attention mechanism, the module is embedded in the residual block structure and named MCSA-ResDNN, and in the model CSA-MResNet proposed in this paper, the attention mechanism is placed between the first convolution layer and the pooling layer and before the last pooling layer for the two streams, respectively. Compare the above two models with the channel spatial attention mechanism and the model without this mechanism. The convolution size in the channel spatial attention mechanism is set to 7. The position comparison results of the channel spatial attention mechanism are shown in Table 3.

From the results in Table 3, it can be seen that the overall *F*1 score of MCSA-ResDNN is increased by 0.7% compared to MResDNN-37 without the channel spatial attention mechanism. The *F*1 score on the PVC category is increased by 10.8%; almost all the average indicators are higher than MResDNN-37. It proves that using the channel spatial attention mechanism can improve performance to a certain extent. The comparison of the results from the different embedding positions of the channel spatial attention mechanism shows that the *F*1 scores of almost all categories of CSA-MResNet are better than MCSA-ResDNN, and the *F*1 scores on the SA category are increased by 1.2%. The *F*1 score of the PVC category has increased by 16.2%. From the above results, it can be seen that CSA-MResNet is the best model in the comprehensive index *F*1 score among the above models. From the model point of view, CSA-MResNet which adds channel spatial attention mechanism to the first two ends of multiscale residual network can pay more attention to more important channels and more important data fragments, while the MCSA-ResDNN which adds channel spatial attention mechanism to a multiscale residual network has better performance than MResDNN-37 which does not add attention mechanism. However, the channel spatial attention mechanism added to the residual structure destroys the performance of the original residual connection to a certain extent, resulting in the model ignoring the information of identity connection in learning and training, thus reducing the learning ability of the model. Therefore, the CSA-MResNet model with channel spatial attention mechanism added to both ends of multiscale residual network performs best.

#### 4.4.4. Other Database Generalization Verification

There are many deep learning methods for intelligent ECG classification, but most previous studies used only one database to verify the results, and there is no independent cross-validation method. Generalization is the difficulty of traditional deep learning [43]. In the actual clinical environment, the ECG data obtained by different collection devices are different, and the ECG data contain a variety of abnormal information about the human body. Whether a single database ECG can cover all ECG features is questionable, so generalization is worth analyzing.

In this work, we verify the CSA-MResNet deep learning model on the HF-challenge testA, use the same network structure and parameter test as Section 3.2, select the corresponding 9 diseases from the database, expand it to 12-lead ECG data according to equation (6), and test it on the dataset with the trained model. The results are shown in Table 4.

The results in Table 4 show that the CSA-MResNet model has lower average *F*1 scores, less than 60% in all, and lower generalization performance on the SA, TWFL, and APB categories. This may be because the ECG data for these categories are more complex or because of the small amount of experimental data, illustrating that these categories in the CCDD cannot contain all the abnormal information. We can think that if samples of the abovementioned poor performance diseases are collected from other databases, and the HF-challenge dataset is generalized and verified after multidatabase training, the performance of the model on these types can be improved. But the mean *F*1 scores on the categories SB, ST, CRBBB, and AF were all greater than 90% and comparable to those tested on the CCDD. Finally, on average metrics, both Acc and Rec were lower than results on the CCDD, and Spe and Pre were higher than the CCDD average results. The average *F*1 score of 85.8% on this dataset and the average *F*1 score obtained on the CCDD do not differ much, demonstrating a certain generalization of the model proposed in this work.

#### 4.4.5. Comparison with Previous Studies

Table 5 shows the contrasting results of different classification methods on the clinical CCDD between our method and others. The results show that CSA-MResNet end-to-end deep learning model is able to provide better classification performance and compare with other works discussed in this paper. The *F*1 score for multilabel classification of the final model was 88.2%, which provided a better method for multilabel classification.

Previous studies in the CCDD [32, 45], respectively, used CBRNN and LCNN models to conduct two normal and abnormal classifications on the database. Literature [44] used ensemble learning methods to identify both normal and abnormal categories, and [46] used heart rate to screen the ECGs and then use LCNN to conduct two normal and abnormal classifications. Literature [47] used ResNet50 for two classifications with a classification accuracy of 89.43%, demonstrating that the ResNet had a good performance on the CCDD. The above research works performed normal and abnormal classifications on the CCDD, and the classification performance indexes were expressed by the accuracy, and it can be seen that the best result was 89.43%, while literature [24] is the only experiment in a comparative research work using the CCDD for multilabel ECG classification. For multilabel classification experiments, it is more reasonable to use the average *F*1 score as an evaluation index due to the problem of sample imbalance. Literature [24] used the integrated multilabel classification model to achieve a final *F*1 score of 75.2% in 7 ECG categories. This work uses the CSA-MResNet model to classify 9 ECG multilabels, and the *F*1 score of this work is 88.2%, indicating that this model is more competitive than the latest methods.

## 5. Conclusion

In order to solve the problem of multilabel classification of clinical ECG, a multiscale residual deep neural network CSA-MResNet model based on the channel spatial attention mechanism for automatic multilabel classification is proposed in this work. The final *F*1 score is 88.2%. The model has a good recognition rate for multilabel ECG classification and provides a feasible analysis method for multilabel ECG classification. This work also verified the model on other HF-challenge testA, and the final *F*1 score was 85.8%, proving that the model is generalizable. However, the experimental data do not include all ECG categories and more experimental data are needed. In the future work, we will pay more attention to this aspect of research.

## Figures and Tables

**Figure 1:** Record CCDD/96833 (0–5000): Atrial premature beats, premature ventricular contraction, and complete right bundle branch block.

**Figure 2:** The architecture for CSA-MResNet.

**Figure 3:** Layer configuration for multiscale residual network.

**Figure 4:** Channel convolution attention mechanism diagram (top (a): channel attention mechanism; bottom (b): spatial attention mechanism).

**Table 1:** The number of 9 disease types used in this work is in different databases.

	CCDD training	CCDD testing	HF-challenge testA
SA	2411	2507	54
SB	2903	2042	724
TWFL	4603	2015	262
ST	2747	1737	357
CRBBB	1892	1056	46
AF	1746	769	121
APB	1714	711	51
I-AVB	1534	634	9
PVC	1158	427	35
Total	17952	10635	1247

**Table 2:** Results of different convolution kernel size models on the CCDD testing (%).

	*F*1					
	MResDNN-37	MResDNN-57	MResDNN-77	MResDNN-79	MResDNN-711	MResDNN-357
SA	86.1	84.9	85.7	85.0	85.6	85.9
SB	93.0	93.2	92.9	93.0	93.2	93.0
TWFL	79.6	79.6	78.8	79.5	78.5	78.2
ST	95.3	95.6	95.6	95.2	95.8	95.5
CRBBB	97.5	95.1	96.6	96.2	95.6	93.8
AF	95.7	96.0	96.0	95.8	94.6	95.9
APB	61.7	60.7	58.3	58.9	59.0	58.4
I-AVB	78.6	78.4	79.1	79.2	76.6	77.6
PVC	60.4	66.6	72.8	75.3	59.0	67.3

Average						
Acc	96.8	96.7	96.8	96.7	96.7	96.7
Spe	98.6	98.5	98.6	98.5	97.6	98.5
Pre	89.7	88.8	90.3	88.6	83.1	88.9
Rec	84.0	84.2	83.5	84.6	89.4	83.6
*F*1	86.8	86.5	86.7	86.5	86.1	86.2

**Table 3:** Results of different positions of channel spatial attention mechanism on the CCDD testing (%).

	*F*1		
	MResDNN-37	MCSA-ResDNN	CSA-MResNet
SA	86.1	86.9	87.3
SB	93.0	93.3	93.0
TWFL	79.6	79.7	80.5
ST	95.3	95.7	95.8
CRBBB	97.5	95.9	96.4
AF	95.7	95.6	96.9
APB	61.7	69.9	69.9
I-AVB	78.6	78.6	80.2
PVC	60.4	71.2	76.6

Average			
Acc	96.8	97.0	97.1
Spe	98.6	98.6	98.7
Pre	89.7	89.8	90.6
Rec	84.0	85.4	85.9
*F*1	86.8	87.5	88.2

**Table 4:** The classification performance of the proposed model is verified in HF-challenge testA (%).

	Acc	Spe	Pre	Rec	*F*1
SA	93.7	94.6	37.9	72.2	49.7
SB	93.4	100	100	88.7	94.0
TWFL	84	99.7	95.7	25.2	39.9
ST	99.4	100	100	97.8	98.9
CRBBB	99.8	99.9	97.8	97.8	97.8
AF	99.8	99.9	99.2	99.2	99.2
APB	97.0	99.6	79.2	37.3	50.7
I-AVB	99.6	99.9	83.3	55.6	66.7
PVC	98.6	99.8	87.0	57.1	69.0
Average	96.1	99.1	94.0	78.9	85.8

**Table 5:** Comparison results of different research work on the CCDD.

Literature	ECG categories	Classifier	Performance
[32]	2	CBRNN	Spe = 76.32% Se = 75.52% Acc = 87.69%

[44]	2	Ensemble deep learning	Spe = 86.86 ± 3.51% Se = 80.23 ± 4.49% Acc = 84.84 ± 1.82%

[45]	2	LCNN	Spe = 83.84% Se = 83.43% Acc = 83.66%

[46]	2	Heart rate and LCNN fuse	Spe = 84.45% Se = 85.19% Acc = 84.77%

[47]	2	ResNet50	Spe = 91.63% Se = 87.73% Acc = 89.43%

[24]	7 multilabel	Ensemble multilabel classification model	Se (Rec) = 71.6% Acc = 75.2% Pre = 80.8% *F*1 = 75.2%

This work	9 multilabel	CSA-MResNet	Spe = 98.7% Se (Rec) = 85.9% Acc = 97.1% Pre = 90.6% *F*1 = 88.2%

## Data Availability

The data used to support the findings of this study are included within the article. Further data can be requested from the corresponding author.
